# Topical Treatment with Xiaozheng Zhitong Paste (XZP) Alleviates Bone Destruction and Bone Cancer Pain in a Rat Model of Prostate Cancer-Induced Bone Pain by Modulating the RANKL/RANK/OPG Signaling

**DOI:** 10.1155/2015/215892

**Published:** 2015-01-27

**Authors:** Yanju Bao, Yebo Gao, Maobo Du, Wei Hou, Liping Yang, Xiangying Kong, Honggang Zheng, Weidong Li, Baojin Hua

**Affiliations:** ^1^Department of Oncology, Guang'anmen Hospital, China Academy of Chinese Medical Sciences, Beixiange 5, Xicheng District, Beijing 100053, China; ^2^Beijing University of Chinese Medicine, Beijing North Third Ring Road No. 11, Chaoyang District, Beijing 100029, China; ^3^Institute of Chinese Materia Medica, China Academy of Chinese Medical Sciences, Nanxiaojie, Dongzhimen District, Beijing 100700, China; ^4^Department of Nephrology, Guang'anmen Hospital, China Academy of Chinese Medical Sciences, Beixiange 5, Xicheng District, Beijing 100053, China

## Abstract

To explore the effects and mechanisms of Xiaozheng Zhitong Paste (XZP) on bone cancer pain, Wistar rats were inoculated with vehicle or prostate cancer PC-3 into the tibia bone and treated topically with inert paste, XZP at 15.75, 31.5, or 63 g/kg twice per day for 21 days. Their bone structural damage, nociceptive behaviors, bone osteoclast and osteoblast activity, and the levels of OPG, RANL, RNAK, PTHrP, IGF-1, M-CSF, IL-8, and TNF-*α* were examined. In comparison with that in the placebo group, significantly reduced numbers of invaded cancer cells, decreased levels of bone damage and mechanical threshold and paw withdrawal latency, lower levels of serum TRACP5b, ICTP, PINP, and BAP, and less levels of bone osteoblast and osteoclast activity were detected in the XZP-treated rats (*P*<0.05). Moreover, significantly increased levels of bone OPG but significantly decreased levels of RANL, RNAK, PTHrP, IGF-1, M-CSF, IL-8, and TNF-*α* were detected in the XZP-treated rats (*P*<0.05 for all). Together, XZP treatment significantly mitigated the cancer-induced bone damage and bone osteoclast and osteoblast activity and alleviated prostate cancer-induced bone pain by modulating the RANKL/RANK/OPG pathway and bone cancer-related inflammation in rats.

## 1. Introduction

Cancer pain is reported to be experienced by 75%–90% of late stage metastatic cancer patients [1]. Cancer-induced bone pain (CIBP) is the most common type of cancer pain and is often debilitating and intractable, affecting the quality of life and functional status in cancer patients [2, 3]. Bone cancer pain is not a single entity but is a combination of background and breakthrough pain, which is defined as “a transitory exacerbation of pain experienced by the patient who has relatively stable and adequately controlled baseline pain” [2]. Currently, there are many therapeutic options available for the alleviation of bone cancer pain and they include external beam radiotherapy, opioid analgesia, nonsteroidal anti-inflammatory drugs (NSAIDs), bisphosphonates, local surgery, and anaesthetic techniques [4]. However, each of these treatment options is accompanied by limitations of less effectiveness and severe effects [4–9]. Hence, control of bone cancer pain will be of great significance in management of patients with bone cancer.

According to traditional Chinese medicine (TCM) theory, cancer pain is the result of tumor-caused stagnation and insufficiency of Qi and blood flow in the body. Thus the main therapeutic goals are to promote Qi and activate blood by softening hard lumps, dispelling nodes, and warming the channels [10]. Our previous study has demonstrated that herbal analgesic paste, Xiaozheng Zhitong Paste (XZP) containing six herbs of Xuejie (Dragon's blood), Yanhusuo (*Corydalis rhizoma*), Ruxiang (Olibanum), Moyao (Myrrha), Qingdai (Natural Indigo), and Bingpian (Borneolum Syntheticum), significantly alleviated cancer pain including bone cancer pain in patients with middle/late stage cancer [11]. However, the mechanisms underlying action of XZP in alleviating bone cancer pain have not been systemically explored. In advanced medicine, the development of bone cancer pain has been attributed to cancer-related bone destruction, reactive muscle spasm, cancer-related inflammation, and release of inflammatory mediators as well as increased concentrations of calcium [2]. During the process of bone cancer pain, aberrant activation of osteoclasts and compensatively increased osteoblast activity contribute to the bone structural damage and are positively regulated by the receptor activator of nuclear factor-*κ*B (RANK) ligand (RANKL) [12], but negatively regulated by osteoprotegerin (OPG). Furthermore, the bone formation and resorption are also regulated by the parathyroid hormone related proteins (PTHrP) and insulin-like growth factor 1- (IGF-1-) related signaling [13, 14]. Accordingly, the levels of serum tartrate-resistant acid phosphatase 5b (TRACP5b), carboxy-terminal pyridinoline cross-linked telopeptide of type I collagen (ICTP), procollagen type I amino-terminal propeptide (PINP), and bone alkaline phosphates (BAP) have been used to estimate bone destruction in patients with bone metastatic cancers, such as prostate cancer [15–17]. In addition, bone cancer can cause inflammation and produce inflammatory cytokines, such as interleukin 8 (IL-8), tumor necrosis factor- (TNF-) *α*, and macrophage colony-stimulating factor (M-CSF), which feedback induce bone damage and pain [12, 18, 19]. It is unclear whether and how XZP treatment can inhibit cancer invasion in the bone and related bone damage as well as osteoclast and osteoblast activity. Furthermore, it is still unknown on whether and how XZP treatment can modulate the activation of the RANKL/RANK/OPG signaling and the expression of bone metabolic regulators and inflammatory mediators.

The aim of this study was to evaluate the effects of XZP and to explore the mechanisms underlying its action in alleviating bone cancer pain. We employed a rat model of bone prostate cancer pain to test the hypothesis that XZP can alleviate bone cancer pain by modulating the RANKL/RANK/OPG signaling and the expression of bone metabolic regulators of PTHrP and IGF-1 and inflammatory mediators of IL-8, M-CSF, and TNF-*α* in the bone of rats.

## 2. Materials and Methods

### 2.1. Composition and Preparation of XZP

XZP was composed of six traditional Chinese medicines, which were purchased from Tong-Ren-Tang (Beijing, China) and authenticated by Professor Hu Shilin, Institute of Chinese Materia Medica, China Academy of Chinese Medical Sciences. The basic pharmacological functions of these Chinese medicines are illustrated in Table 1. All the components of XZP were dried and homogenized to fine powders. To prepare the XZP, individual powdered medicine (950 g) was extracted twice with 70% ethanol (1 : 5 w/v) for 1–1.5 h each. The extracts were filtrated and concentrated to 1 g per 3.59 g (crude herbs), followed by being stored at −20°C. The extracts were mixed with cataplasm matrix to generate a proper concentration of XZP before use in vivo.

### 2.2. High Performance Liquid Chromatography

To determine the potential components, the XZP was prepared and analyzed by high performance liquid chromatography (HPLC) using >98% purity of the standards of tetrahydropalmatine, imperatorin, isoimperatorin, coptisine, and palmatine chloride (in methanol) that were purchased from the National Institute for Food and Drug Control (Beijing, China). Methanol and acetonitrile (HPLC grade, Fisher Scientific, New Jersey, USA) and pure water (Wahaha Group, China) were used for HPLC analysis. All other chemicals were of analytical grade. The solutions were filtered through 0.45 *μ*m membranes and subjected to analysis at 280 nm using an Agilent Zorbax Eclips XDB C18 column (250 × 4.6 mm, 4.5 *μ*m) on a Waters HPLC system (Waters Corporation, USA) equipped with 2487 pump, an UV detector, an Empower 2 system controller, and a waters 717 plus autosampler at 30°C. Samples at 10 *μ*L were injected and acetonitrile-methanol-water-triethylamine (24 : 32 : 44 : 0.5) at a flow-rate of 1.0 mL per min was used at the mobile phase. According to the chromatographic characteristics of these standard compounds, the peak areas of individual compounds in the samples were used for determining the contents of these compounds and expressed as the percent.

### 2.3. Animals

Female Wistar rats weighing 150–180 g were from the Department of Experimental Animal Sciences, Peking University Health Science Center (Beijing, China). Individual rats were housed in specific pathogen free (SPF) facility at 24 ± 1°C on a cycle of 12/12 h light/dark and free access to food and water. All experiments were carried out in accordance with the guidelines of the International Association for the Study of Pain [20] and approved by the Animal Care and Use Committee of China Academy of Chinese Medical Sciences.

### 2.4. Cell Preparation and Bone Cancer Pain Model

Prostate cancer PC-3 cells were prepared and bone cancer pain model were established, as our previous report [21]. Briefly, individual rats were anesthetized intraperitoneally (i.p) with sodium pentobarbital (45 mg/kg) and the left tibia of individual rats was exposed. The left tibia of individual rats was injected with 10^5^ PC-3 cells in 10 *μ*L Hank's solution and the injection site was covered by bone wax, followed by closing the wound. A group of rats (*n* = 10) received the same surgery and the same volume of vehicle injection and served as the Sham controls. All rats were subjected to the same postoperational cares.

### 2.5. Treatment and Groups

The Sham control rats were treated topically with the inert paste as the control (*n* = 10 per group). The bone cancer-bearing rats were randomly and treated topically with the inert paste as the placebo, the XZP at 15.75 g/kg (as the low dose), 31.5 g/kg (medium dose), or 63 g/kg (high dose) evenly applied on the skin of tumor-bearing tibias, covered with gauze and a layer of plastic film, sealed, and fixed with desensitized adhesive plaster twice a day at 8:00 AM and 20:00 PM for consecutive 21 days beginning one day after Walker 256 cell inoculation [11].

### 2.6. Radiological Analysis

The cancer-related osteolytic lesions in the tibia of individual rats were examined by X-ray radiology at 21 days after the inoculation. The rats were anaesthetized and exposed to X-ray (Emerald 125) at 40 KVP for 1/20 s, followed by the development of X-ray film (Henry Schein blue sensitive film) using a film developer (Konica SRX-101). The radiological score was calculated according to Stewart's radiological score [22]: 0: normal bone structure with no sign of deterioration; 1: minor loss of medullary bone; 2: substantial loss of medullary bone with erosion of cortical bone; and 3: substantial loss of medullary bone with major cortical destruction of the proximal epiphysis.

The tibias were scanned by micro-CT and reconstructed with 8 *μ*m isotropic voxel size on a micro-CT system (eXplore Locus SP, GE Medical Systems). The reconstructed 3D imagines of femurs were analyzed using Microviewer (GE Medical Systems), as described previously [23]. Micro-CT is used to measure several histomorphometric variables including bone volume (BV), total volume (TV), and bone volume fraction (BV/TV) [24].

### 2.7. Mechanical Threshold and Paw Withdrawal Latency

The effects of treatment with XZP on the spontaneous nocifensive behaviors of the different groups of rats were tested for the mechanical threshold and paw withdrawal latency (PWL) in a blinded manner, as our previous description [21, 25, 26]. In brief, individual rats were placed in an inverted plastic chamber on the glass surface of the Paw Thermal Stimulator System (UCSD, San Diego) for 30 min before the test. Mechanical hyperalgesia was measured using a single rigid filament attached to a handheld transducer (automatic plantar analgesia tester; Institute of Biomedical Engineering, Chinese Academy of Medical Science, Tianjin, China). Animals were acclimated to their surroundings for 10 min daily for three consecutive days in a plexiglass box on a metal grid surface prior to testing. On the testing days, rats were allowed to acclimate for 5–10 min. A rigid filament was pressed perpendicularly against the medial plantar surface of the hind paw with an increasing force. Brisk paw withdrawal or paw flinching accompanied by head turning, biting, and/or licking upon application of an increasing force was considered as a positive response. The paw withdrawal threshold (PWT) was defined as the minimal force (g) required to evoke the cited positive responses. Each hind paw of rats was tested three times and the data were averaged. The interval between consecutive tests of the same paw was 5 min. The same procedure was performed on days 3, 6, 9, 12, 15, 18, and 21 after tumor inoculation. Each hind paw of rats was stimulated with a focused beam of radiant heat using an analgesiometer (37360, Ugo Basile, Italy) underneath the glass surface. When the paw was withdrawn from the stimulus the PWL was automatically recorded to the nearest 0.1 s. The intensity of stimuli was adjusted to generate an average baseline PWL of approximately 10.0 s in naive animals. The maximum stimulation was controlled <20 s to prevent potential tissue damage. Paws were alternated randomly to preclude “order” effects. Individual rats were subjected to four tests with a 5 min interval before surgery and 2, 5, 8, 11, 14, 17, and 20 days after inoculation in a blinded manner. The mean PWL was calculated for each time point in individual rats.

### 2.8. Histological Evaluation

The rats were deeply anesthetized by pentobarbital and transcardially perfused with saline on day 21 after inoculation (*n* = 10 per group). The left tibia from each animal was dissected, fixed in 10% formalin overnight, decalcified in 15% EDTA-PBS for 7 days, and paraffin-embedded. The tissue sections (6 *μ*m) were stained with hematoxylin and eosin (HE). Furthermore, the numbers of osteoclasts and osteoblasts in the regions were identified by the tartrate-resistant acid phosphatase (TRAP) or alkaline phosphatase (AP) staining using the TRAP or AKP staining kits (Nanjing Jiancheng Bioengineering Institute, Nanjing, China), respectively. The numbers of osteoclasts and osteoblasts in 10 sections from each rat were counted under a light microscope (Leica DM 2500) in a blinded manner [25].

### 2.9. Enzyme-Linked Immunosorbent Assay (ELISA)

Peripheral blood samples were collected from individual rats at 0, 7, 14, or 21 days after inoculation and the concentrations of serum tartrate-resistant acid phosphatase 5b (TRACP5b), carboxy-terminal pyridinoline cross-linked telopeptides of type I collagen (ICTP), procollagen type I amino-terminal propeptide (PINP), and bone alkaline phosphatase (BAP) in individual rats were determined by ELISA using the specific kits, according to the manufacturer's instruction (Thermo Scientific, Hudson, NH, USA). The limitation of detection for TRACP5b, ICTP, PINP, and BAP was 0.078 mIU/mL, 25 ng/mL, 18.75 pg/mL, and 25 U/L, respectively.

### 2.10. Quantitative RT-PCR

Total RNA was extracted from individual rat tibias using the TRIzol reagent and reversely transcribed to cDNA using the first-strand cDNA synthesis kit (Invitrogen). The relative levels of target gene mRNA transcripts were determined by quantitative RT-PCR using the SYBR Green system and specific primers on the LightCycler system (Roche). The sequences of primers are shown in Table 2. The PCR amplification was performed in triplicate at 95°C for 10 minutes and was subjected to 40 cycles of 95°C for 15 s and 60°C for 30 s. The relative levels of each gene to GAPDH mRNA transcripts were calculated.

### 2.11. Western Blot Assay

Total tibia proteins were extracted from individual rats by sonication in RIPA buffer containing protease inhibitors (Roche). After quantification of protein concentrations using the BCA protein assay kit (Thermo Scientific, Rockford, IL), the protein samples (20 *μ*g/lane) were separated by sodium dodecyl sulfate polyacrylamide gel electrophoresis (SDS-PAGE) and transferred onto polyvinylidene difluoride (PVDF) membranes (Millipore). After being blocked with 5% fat-free dry milk, the membranes were incubated with anti-OPG (ab73400), anti-GAPDH (6C5, ab8245), anti-IL-8 (ab7747), anti-PTHrP (ab85205), anti-M-CSF (ab99109), anti-IGF1 antibody (ab36532), anti-TNF-*α* (ab66579), anti-RANKL (EPR4999, ab124797, Abcam, Cambridge, MA, USA), and anti-RANK (H-300, sc-9072, Santa Cruz Biotechnology), respectively. The bound antibodies were detected using a horseradish peroxidase- (HRP-) conjugated secondary antibody and visualized by an enhanced chemiluminescence detection system, followed by quantifying using the Image Quant LAS 4000 (GE Healthcare).

### 2.12. Statistical Analysis

Data are expressed as the mean ± standard deviation (SD) and analyzed by two-way repeated ANOVA or by one-way ANOVA, followed by a Newman-Keuls test using SPSS 13.0 statistical software. A *P* value of <0.05 was considered statistically significant.

## 3. Results

### 3.1. HPLC Analysis of XZP

Our previous study has shown that XZP, prepared from six herbs of Xuejie (Dragon's blood), Yanhusuo (*Corydalis rhizoma*), Ruxiang (Olibanum), Moyao (Myrrha), Qingdai (Natural Indigo), and Bingpian (Borneolum Syntheticum), significantly alleviates bone cancer pain in patients with middle/late stage of cancer [11]. To understand the effect of XZP, the major components in the ethanol-extracted XZP were analyzed by HPLC. We found that the XZP contained tetrahydropalmatine (0.0568%), imperatorin (0.0041%), isoimperatorin (0.0122%), coptisine (0.0358%), and palmatine chloride (0.112%, Figure 1).

### 3.2. The Effect of XZP on the Implanted Cancer Growth and Bone Destruction

At 21 days after inoculation, all rats were sacrificed and their tibial bones were examined by X-rad and micro-CT as well as pathology, while there is no radiological change in the tibial bones of the control group of rats (Figure 2(a)). Less degrees of medullary bone loss and the cortical bone erosion were apparent in the rats that had been treated with XZP. Quantitative analysis revealed that the radiological scores in the rats that had been treated with different doses of XZP were significantly less than that of the placebo group (*P* < 0.05 or *P* < 0.01) although they were still significantly higher than that of the healthy controls. Micro-CT examinations indicated that the percentages of bone volume in total volume in the XZP-treated rats were significantly greater than that of the placebo group of rats (*P* < 0.05 or *P* < 0.01, Figure 2(b)) and the effect of XZP on preserving the bone structure appeared to be dose-dependent. In addition, histological examination revealed that while many cancer cells are invaded in the bone tissues of the placebo group of rats the numbers of invaded cancer cells in the bone of the XZP-treated rats were obviously reduced, particularly from the rats that had been treated with a higher dose of XZP (Figure 2(c)). Collectively, treatment with XZP mitigated the cancer invasion into the bone and cancer-related bone destruction in rats.

### 3.3. The Effect of XZP Treatment on the Nociceptive Behaviors in Rats

Bone cancer usually causes severe pain in humans and nociceptive responses in animals. The effects of XZP on bone cancer-related nociceptive behaviors of the PAT and PWL in the different groups of rats were measured longitudinally after inoculation. While similar levels of PWT were observed in the control rats throughout the observation period, the levels of PWT were gradually reduced (Figure 3(a)). In contrast, treatment with different doses of XZP significantly mitigated the mechanical allodynia in a dose and time-dependent manner. A similar pattern of the PWL was observed in the different groups of rats (Figure 3(b)). Hence, treatment with XZP reduced the mechanical and thermal nociceptive behaviors in rats with bone cancer.

### 3.4. The Effect of XZP Treatment on the Levels of Osteoclast and Osteoblast Activity in Bone Cancer Rats

To understand the effect of XZP treatment on the levels of osteoclast and osteoblast activity, the levels of serum TRACP 5b, ICTP, PINP, and BAP in individual rats were measured longitudinally by ELISA. First, there was no significant difference in the levels of serum TRACP5b, ICTP, PINP, and BAP among the different groups of rats before inoculation (Figure 4). Second, the levels of serum TRACP5b, ICTP, PINP, and BAP in the placebo group of rats were significantly higher than that of the control throughout the observation period (*P* < 0.01). In contrast, the levels of serum TRACP5b, ICTP, PINP, and BAP in the XZP-treated rats, particularly for the rats that received a high dose of XZP, were significantly lower than that of the placebo group (*P* < 0.05) although they remained significantly higher than that of the controls (*P* < 0.05).

In parallel, the activity of osteoclasts and osteoblasts in the bone tissues from the different groups of rats was further evaluated by AP and TRAP staining, respectively. There were a few AP+ osteoblasts in the bone sections of the control rats and increased numbers of AP+ osteoblasts were detected in the bone sections of the placebo group of rats, but not obviously in the bone sections from the XZP-treated rats (Figure 5(a)). Quantitative analysis indicated that the numbers of AP+ osteoblasts in the bone sections from the XZP-treated rats were significantly less than that in the placebo rats at 14 and 21 days after inoculation (*P* < 0.05) but remained significantly greater than that in the controls (*P* < 0.05). Furthermore, the numbers of TRAP+ osteoclasts in the XZP-treated rats were significantly greater than that in the controls (*P* < 0.05) but were significantly less than in the placebo group of rats at 7, 14, and 21 days after inoculation (*P* < 0.05, Figure 5(b)). Together, treatment with XZP mitigated the cancer-stimulated osteoclast and osteoblast activity in vivo.

### 3.5. XZP Treatment Modulates the OPG/RANKL/RANK Signaling and Other Bone Regulator Expressions in the Bone of Rats

The bone metabolism is regulated by the OPG/RANKL/RANK signaling, inflammatory mediators, and hormone and IGF-1 [12–14]. To understand molecular mechanisms by which XZP inhibited the cancer-related bone destruction, the relative levels of OPG, RANKL, RANK, IL-8, PTHrP, M-CSF, IGF-1, and TNF-*α* in the bones from the different groups of rats were analyzed by quantitative RT-PCR. The relative levels of OPG mRNA transcripts to control GAPDH in the XZP-treated rats at different time points post inoculation were significantly higher than that in the placebo group (*P* < 0.05, or *P* < 0.01) but were significantly higher than that in the control (*P* < 0.05, Figure 6(a)). In contrast, the relative levels of RANKL, IL-8, PTHrP, M-CSF, IGF-1, and TNF-*α* but not RANK mRNA transcripts in the placebo group at different time points after inoculation were significantly higher than that in the controls (*P* < 0.05 or *P* < 0.01, Figures 6(b)–6(h)), except that there was no significant difference in the relative levels of IGF-1, M-CSF, and TNF-*α* mRNA transcripts between these two groups of rats at earlier time points after inoculation. The relative levels of RANKL, RANK, IL-8, PTHrP, M-CSF, IGF-1, and TNF-*α* mRNA transcripts in the XZP-treated rats were significantly lower than that in the placebo group of rats (*P* < 0.05 or *P* < 0.01), except that the relative levels of IL-8, PTHrP, M-CSF, and TNF-*α* mRNA were higher than that in the placebo group at earlier time points after inoculation.

Further Western blot analysis revealed that in comparison with that in the placebo group of rats, significantly higher levels of OPG and lower levels of RANKL, RANK, IL-8, PTHrP, M-CSF, IGF-1, and TNF-*α* were detected in the bones of the control group of rats (Figure 7). In contrast, the relative levels of OPG in the bones from the XZP-treated rats significantly increased while the relative levels of RANKL, RANK, IL-8, PTHrP, M-CSF, IGF-1, and TNF-*α* in the bones from the XZP-treated rats were significantly reduced (*P* < 0.05, *P* < 0.01, or *P* < 0.001). The modulatory effects of different doses of XZP were dose-dependent in rats. Collectively, these data indicated that XZP treatment modulated the expression of OPG/RANKL/RANK pathway events and other bone metabolic regulators as well as inflammatory mediators in the cancer bones of rats.

## 4. Discussion

In this study, we examined the effects of XZP treatment on the bone prostate cancer nociceptive behaviors and potential mechanisms underlying the action of XZP treatment in a rat model of prostate cancer bone pain. We found that XZP treatment significantly mitigated cancer invasion and bone damage as well as nociceptive behaviors in rats, consistent with our previous findings [11]. Furthermore, we found that XZP treatment significantly reduced the levels of serum TRACP5b, CIPT, PINP, and BAP and the AP+ osteoblasts and TRAP+ osteoclasts in rats, related to that of placebo group, demonstrating that XZP treatment mitigated the bone cancer-induced aberrant activation of osteoclasts and osteoblasts. In addition, we found that XZP treatment upregulated OPG expression but downregulated RANKL, RANK, Il-8, M-CSF, TNF-*α*, PTHrP, and IGF-1 expression in the tibial bones of rats, as compared with that in the placebo group. These data indicated that XZP treatment inhibited the activation of bone cancer-related RANKL/RANK/OPG pathway and inflammation, leading to a reduction in the cancer-related bone destruction and alleviation of bone cancer pain in rats. To the best of our knowledge, this was the first study on the mechanisms underlying the action of XZP. Our findings may provide new insights into understanding the molecular pathogenesis of bone cancer pain and aid in design of new therapies for intervention of bone cancer pain.

Bone cancer pain is associated with bone destruction, which is attributed to aberrant activation of osteoclasts [3, 27, 28]. The functional development of osteoclasts is positively regulated by the RANKL/RANK-related signaling but is negatively regulated by OPG [12, 29]. Furthermore, the activity of osteoclasts is also regulated by the IGF-1-related signaling and PTHrP and other hormones [13–18]. In this study, we found that in comparison with that in the placebo group, XZP treatment significantly mitigated the bone cancer-upregulated RANKL, RANK, PTHrP, IGF-1, IL-8, M-CSF, and TNF-*α* but increased the levels of OPG expression in the tibial bones of rats, accompanied by decreased numbers of osteoclasts and osteoblasts. These data were consistent with previous findings [30–33] and support the notion that the RANKL/RANK/OPG signaling is crucial for the development and progression of bone cancer pain [12, 34–36]. It is likely that bone metastasis of cancer cells recruits inflammatory infiltrates, which secrete inflammatory mediators such as IL-8, TNF-*α*, and M-CSF, and promotes osteoclastogenesis, leading to the bone destruction and bone cancer pain. Hence, the RANKL/RANK/OPG signaling may be a target for the design of new therapies for intervention of bone cancer pain.

Aberrant activation of osteoclasts also compensatively promotes the activity of osteoblasts to balance the bone absorption and formation [12, 35, 37, 38]. We detected high levels of serum PINP and BAP and increased numbers of AP+ osteoblasts in the tibial bones of the placebo group of rats. Indeed, the levels of serum PINP and BAP have been used as biomarkers for evaluating the bone turnover in patients with bone metastatic cancer [15–17]. However, XZP treatment significantly reduced the values of serum TRACP5b and CIPT but also decreased the levels of serum PINP and BAP in rats, further supporting that aberrant activation of osteoclasts enhanced the activity of osteoblasts in the bone cancer rats. Therefore, aberrant activation of osteoclasts should be therapeutic targets for treatment of bone cancer pain [39, 40].

In TCM, tumor-caused stagnation and insufficiency of Qi and blood flow in the body are responsible for the development of bone cancer pain while increase in the Qi and blood flow such as softening hard lumps, dispelling nodes, and warming the channels is crucial for alleviation of bone cancer pain [10]. We found that XZP treatment significantly alleviated the bone cancer-related nociceptive behaviors. Indeed, the herbs in the XZP formula have been used for the control of pain in TCM for many years. Dragon's blood contains cochinchinenin A, cochinchinenin B, and loureirin B and can inhibit the expression of Cox2 and substance P and reduce the levels of intracellular calcium, leading to potent analgesic activity [41, 42]. Yanhusuo (*Corydalis rhizome*) can also significantly inhibit formalin-evoked spontaneous nociceptive responses in rodents [43] and combination of Yanhusuo (*Corydalis rhizome*) and Baizhi (*Angelicae dahuricae*) alleviates pain in a clinical trial [44]. Ruxiang (Olibanum) and Moyao (Myrrha) can also have anti-inflammatory and analgesic activities, respectively [45]. It is possible that these drugs in the XZP synergistically inhibited inflammation and promoted the Qi and blood flow, alleviating bone cancer nociception in rats.

In conclusion, our data demonstrated that XZP treatment significantly reduced cancer invasion, related osteoclast activity, and bone destruction as well as nociceptive behaviors in rats by modulating the RANKL/RANK/OPG signaling and the expression of inflammatory mediators and bone metabolic regulators. Therefore, our findings may provide a new basis for the design of therapies for intervention of bone cancer pain.

## Figures and Tables

**Figure 1:** HPLC analysis of the components of XZP. XZP were extracted with ethanol and the representative active components in the XZP extracts were characterized by HPLC using the standard components of (A) tetrahydropalmatine, (B) imperatorin, (C) isoimperatorin, (D) coptisine, and (E) palmatine chloride. Data are representative chromatographic histograms at 280 nm of XZP (a), characterized profile (UV chromatograms at 280 nm) of the standard compounds (a), XZP ethanol-extracts (b), and blank (c) from three independent experiments. (d) The structures of standard compounds.

**Figure 2:** XZP treatment reduces the cancer-induced bone damage in rats. At 21 days after inoculation, the tibial bone structure and damage in the individual rats were characterized by X-rad and micro-CT and quantitatively analyzed. Subsequently, their tibial bone sections were stained with HE. Data are representative images of individual groups of rats (*n* = 10 per group). (a) Radiographs of the bone structure and tumor invasion. (b) 3D micro-CT images of the tibias. (c) HE analysis of the cancer bone tissues (magnification ×400). Low dose, medium dose, and high dose. The rats were treated with low, medium, or high dose of XZP. (^**^ *P* < 0.01 versus the control group; ^#^ *P* < 0.05 versus the placebo group; ^**^ *P* < 0.01 versus placebo group).

**Figure 3:** XZP treatment mitigates the bone cancer-related nociceptive behaviors in rats. The mechanical allodynia and paw withdrawal latency of individual rats before and at the indicated time points after inoculation were measured. Data are expressed as the means ± SD of individual groups of rats (*n* = 10 per group). (a) The changes in the mechanical allodynia. (b) The changes in thermal hyperalgesia. ^*^ *P* < 0.05, ^**^ *P* < 0.01, ^***^ *P* < 0.001 versus the control group; ^#^ *P* < 0.05 versus the placebo group.

**Figure 4:** XZP treatment modulates the levels of serum TRACP5b, ICTP, PINP, and BALP in rats. The levels of serum TRACP5b, ICTP, PINP, and BALP in individual rats were analyzed at the indicated time points before and after prostate cancer cell inoculation. Data are expressed as the means ± SD of individual groups of rats (*n* = 10 per group) from three separated experiments. (a) The levels of serum TRACP5b. (b) The levels of serum ICTP. (c) The levels of serum PINP. (d) The levels of serum BAP. ^*^ *P* < 0.05 versus the control group; ^#^ *P* < 0.05 versus the placebo group.

**Figure 5:** Histological evaluation of osteoblast and osteoclast activity and macrophage infiltration. The numbers of osteoblasts and osteoclasts in the cancer-invaded tibial bones of individual groups of rats were characterized by AP and TRAP-enzymatic staining, respectively. The yellow-brown staining represents AP+ osteoblasts or TRAP+ osteoclasts, respectively. Data are representative images (magnification ×400) and are expressed as the means ± SD of individual groups of rats (*n* = 10 per group) from three separated experiments. (a) Characterization of osteoblasts; (b) characterization of osteoclasts. ^*^ *P* < 0.05 versus the control group; ^#^ *P* < 0.05 versus the placebo group.

**Figure 6:** Quantitative RT-PCR analysis of the relative levels of target gene mRNA transcripts in the tibial bones of individual groups of rats. The relative levels of OPG, RANKL, RANK, IL-8, PTHrP, M-CSF, IGF-1, and TNF-*α* mRNA transcripts to the control GAPDH in the tibial bones of individual rats at the indicated time points were determined by quantitative RT-PCR. Data are expressed as the means ± SD of individual groups of rats (*n* = 10 per group) from three separated experiments. (a) The levels of OPG mRNA transcripts; (b) the levels of RANKL mRNA transcripts; (c) the levels of RNAK mRNA transcripts; (d) the levels of IL-8 mRNA transcripts; (e) the levels of PTHrP mRNA transcripts; (f) the levels of M-CSF mRNA transcripts; (g) the levels of IGF-1 mRNA transcripts; (h) the levels of TNF-*α* mRNA transcripts. ^*^ *P* < 0.05 versus the control group; ^#^ *P* < 0.05 versus the placebo group.

**Figure 7:** Western blot analysis of the relative levels of OPG, RANKL, RANK, IL-8, PTHrP, M-CSF, IGF-1, and TNF-*α* expression in the tibial bones of individual groups of rats. The relative levels of OPG, RANKL, RANK, IL-8, PTHrP, M-CSF, IGF-1, and TNF-*α* expression in the tibial bones of individual groups of rats at the indicated time points were determined by Western blot assays. Data are representative images and are expressed as the means ± SD of individual groups of rats (*n* = 10 per group) from three separated experiments. (a) Western blot analysis; (b) quantitative analysis; ^**^ *P* < 0.01, ^***^ *P* < 0.001 versus the control group; ^#^ *P* < 0.05 versus the placebo group.

**Table 1:** Composition of XZP.

Pharmaceutical name	Botanical source/family	Part used	Traditional actions/uses	Amount (g)
Dragon's blood	*Daemonorops* *Draco Bl. *	Dried resin	Calms pain, promotes Qi and moves blood, and promotes circulation in the collaterals	10
*Corydalis rhizoma*	*Corydalis yanhusuo W.T.Wang *	Dried rhizome	Calms pain, promotes Qi and moves blood, and promotes circulation in the collaterals	50
Olibanum	*Boswellia carterii Birdw.* *Boswellia bhaw-dajiana Birdw *	Dried resin	Calms pain, moves blood, and promotes circulation in the collaterals	50
Myrrha	*Commiphora myrrha Engl.* *Commiphora molmol Engl. *	Dried resin	Calms pain, moves blood, and promotes circulation in the collaterals	50
Borneolum Syntheticum	—	—	Calms pain	20
Natural Indigo	*Baphicacanthus cusia(Nees) Bremek*. *Polygonum tinctorium Ait.* *Isatis indigotica Fort. *	Dried stem or dried leaves	Anticancer, clearing away heat and toxic material	10

**Table 2:** The sequences of primers.

Target gene	Primers sequences		Size (bp)
OPG	Forward	5′-TTCTAGGCAAGTTGACCGTTAGC-3′	81
	Reverse	5′-TACCCCTGCTTGTCTAGCCAA-3′	

RANKL	Forward	5′-CACAGCGCTTCTCAGGAGTT-3′	101
	Reverse	5′-GATGGTGAGGTGAGCAAACG-3′	

RANK	Forward	5′-CCAGGAGAGGCATTATGAGCA-3′	94
	Reverse	5′-ACTGTCGGAGGTAGGAGTGC-3′	

IL8	Forward	5′-CATTAATATTTAACGATGTGGATGCGTTTCA-3′	76
	Reverse	5′-GCCTACCATCTTTAAACTGCACAAT-3′	

PTHrP	Forward	5′-GGGATCAAACTGTCTCCCCAG-3′	171
	Reverse	5′-AACAGAGTCAGCAGCACCAAG-3′	

M-CSF	Forward	5′-AGCAGGAGTATCACCGAGGA-3′	220
	Reverse	5′-TATCTCTGAAGCGCATGGTG-3′	

IGF-1	Forward	5′-GCTCTTCAGTTCGTGTGTGGA-3′	133
	Reverse	5′-GCCTCCTTAGATCACAGCTCC-3′	

TNF-*α*	Forward	5′-CAGGCGGTGCCTATGTCTC-3′	89
	Reverse	5′-CGATCACCCCGAAGTTCAGTAG-3′	

GAPDH	Forward	5′-CCCCCAATGTATCCGTTGTG-3′	118
	Reverse	5′-TAGCCCAGGATGCCCTTTAGT-3′	
